# Triazole Fungicides Can Induce Cross-Resistance to Medical Triazoles in *Aspergillus fumigatus*

**DOI:** 10.1371/journal.pone.0031801

**Published:** 2012-03-01

**Authors:** Eveline Snelders, Simone M. T. Camps, Anna Karawajczyk, Gijs Schaftenaar, Gert H. J. Kema, Henrich A. van der Lee, Corné H. Klaassen, Willem J. G. Melchers, Paul E. Verweij

**Affiliations:** 1 Department of Medical Microbiology, Radboud University Nijmegen Medical Center, Nijmegen, The Netherlands; 2 Center for Molecular and Biomolecular Informatics, Nijmegen Center for Molecular Life Sciences, Nijmegen, The Netherlands; 3 Nijmegen Institute for Infection, Inflammation, and Immunity (N4i), Radboud University Nijmegen, Nijmegen, The Netherlands; 4 Department of Medical Microbiology and Infectious Diseases, Canisius Wilhelmina Hospital, Nijmegen, The Netherlands; 5 Plant Research International, Wageningen University, Wageningen, The Netherlands; Albert Einstein College of Medicine, United States of America

## Abstract

**Background:**

Azoles play an important role in the management of *Aspergillus* diseases. Azole resistance is an emerging global problem in *Aspergillus fumigatus*, and may develop through patient therapy. In addition, an environmental route of resistance development has been suggested through exposure to 14α-demethylase inhibitors (DMIs). The main resistance mechanism associated with this putative fungicide-driven route is a combination of alterations in the *Cyp51A*-gene (TR_34_/L98H). We investigated if TR_34_/L98H could have developed through exposure to DMIs.

**Methods and Findings:**

Thirty-one compounds that have been authorized for use as fungicides, herbicides, herbicide safeners and plant growth regulators in the Netherlands between 1970 and 2005, were investigated for cross-resistance to medical triazoles. Furthermore, CYP51-protein homology modeling and molecule alignment studies were performed to identify similarity in molecule structure and docking modes. Five triazole DMIs, propiconazole, bromuconazole, tebuconazole, epoxiconazole and difenoconazole, showed very similar molecule structures to the medical triazoles and adopted similar poses while docking the protein. These DMIs also showed the greatest cross-resistance and, importantly, were authorized for use between 1990 and 1996, directly preceding the recovery of the first clinical TR_34_/L98H isolate in 1998. Through microsatellite genotyping of TR_34_/L98H isolates we were able to calculate that the first isolate would have arisen in 1997, confirming the results of the abovementioned experiments. Finally, we performed induction experiments to investigate if TR_34_/L98H could be induced under laboratory conditions. One isolate evolved from two copies of the tandem repeat to three, indicating that fungicide pressure can indeed result in these genomic changes.

**Conclusions:**

Our findings support a fungicide-driven route of TR_34_/L98H development in *A. fumigatus*. Similar molecule structure characteristics of five triazole DMIs and the three medical triazoles appear the underlying mechanism of cross resistance development. Our findings have major implications for the assessment of health risks associated with the use of triazole DMIs.

## Introduction

*Aspergillus fumigatus* is the most frequent cause of *Aspergillus* diseases in humans, which include allergic syndromes, aspergilloma and chronic or acute invasive aspergillosis. Antifungal agents of the azole class play a prominent role in the management of *Aspergillus* diseases. Three medical triazoles, itraconazole, voriconazole and posaconazole, are clinically licensed for the prevention and treatment of *Aspergillus* diseases [1]. It has become apparent that *A. fumigatus* can develop resistance to the medical triazoles. Azole resistance is commonly due to mutations in the *cyp51A*-gene, encoding the target enzyme of antifungal azoles, and both preclinical evidence and clinical experience suggests that reduced *in vitro* susceptibility is associated with increased probability of failure to azole therapy [2]–[4]. Azole resistance may develop during azole therapy, which has been primarily reported in patients with aspergilloma or other *Aspergillus* cavities that received long-term azole therapy [5]. This route of resistance development is characterized by recovery of azole-resistant *A. fumigatus* isolates exclusively from patients receiving azole therapy and by a high diversity of resistance mechanisms. Sometimes multiple resistance mechanisms were found in different *A. fumigatus* colonies recovered from a single patient [5]. The morphotype of *A. fumigatus* appears to be important as the fungus commonly sporulates in cavities, thus creating spores that harbor Cyp51A-mutations [7].

In the Netherlands, we observed azole resistance in *A. fumigatus* isolates from azole-naïve patients and in patients with invasive aspergillosis, which is characterized by hyphal growth in the absence of asexual reproduction. One explanation for this observation could be that a second route of resistance development may exist through environmental exposure of *A. fumigatus* to 14α-demethylase inhibitors (DMIs) [4], [6], [7]. DMIs are abundantly used for crop protection against phytopathogenic molds, for prevention of spoilage post harvest and for preservation of materials. Evidence that supports such a route of resistance development is the dominance of a single resistance mechanism in over 90% of Dutch azole-resistant *A. fumigatus* isolates, recovered from epidemiologically unrelated patients [6]–[8]. This mechanism consists of a 34-bp insertion in the promoter region of the *cyp51A* gene combined with a substitution at codon 98 of leucine to histidine (TR_34_/L98H) [9]. TR_34_/L98H isolates were cultured from patients that were azole-naïve as well as those with previous azole exposure, and were also recovered from the environment [10]. Genetic analysis showed clustering of clinical and environmental TR_34_/L98H isolates compared to wild type controls [6], [10]. TR_34_/L98H isolates exhibit a multi-azole-resistant phenotype and azole-resistant invasive aspergillosis was associated with a high mortality rate of 88% [8], [11]. In the Netherlands the first TR_34_/L98H isolate was cultured in 1998 and since then the prevalence of clinical isolates harboring TR_34_/L98H has increased over time [6], [8].

Theoretically there are significant risks associated with the environmental route of resistance development in fungi. First there is the potential of migration of the resistance trait through sexual or asexual reproduction. It has been shown for phytopathogens that resistance mechanisms may develop locally and subsequently spread across countries [12]. There are early indications that suggest that migration is occurring in TR_34_/L98H as isolates harboring this resistance mechanism have now been reported in other European countries [13], and more recently in azole-resistant isolates in China [14]. The other risk of the environmental route of resistance development is the emergence of multiple resistance mechanisms over time due to continued azole pressure. There are recent reports that indicate that in addition to TR_34_/L98H other ‘environmental’ resistance mechanisms may be emerging [15], [16].

Therefore, it is of great importance to explore the relationship between the use of DMIs and the emergence of TR_34_/L98H in *A. fumigatus* as this may enable effective measures to be taken that prevent further increase of TR_34_/L98H isolates or of the emergence of new resistance mechanisms. The aim of our current research was to determine if route of TR_34_/L98H development could have been fungicide driven. Our hypothesis was that cross-resistance could develop if DMIs and medical triazoles share similar molecule characteristics. This was investigated through molecule alignment and docking studies using a homology model of the CYP51A protein. Furthermore, temporal relationships between DMI exposure and TR_34_/L98H emergence were investigated. Finally, we investigated if the TR_34_/L98H substitutions could be induced through DMI-exposure under laboratory conditions. We were able to identify five triazole DMIs that exhibit highly similar molecule characteristics to medical triazoles and could have caused the emergence of TR_34_/L98H in *A. fumigatus*.

## Methods

### Susceptibility testing

A collection of 25 clinical wild type *A. fumigatus* isolates, 25 clinical azole-resistant TR_34_/L98H isolates, 17 environmental wild type isolates, and 13 environmental TR_34_/L98H isolates were selected for investigation of the *in vitro* activity of fungicides. In addition, two clinical isolates were included that have a tandem repeat as underlying resistance mechanism similar to TR_34_/L98H: one isolate harbored a 53-bp tandem repeat and the other a 46-bp tandem repeat in combination with two substitutions in the *cyp51A*-gene at codons 121 and 289. Finally, four isolates were included that had a resistance mechanism that arose through azole therapy, consisting of point mutations in the *cyp51A*-gene. All isolates were previously identified by sequencing parts of the β-tubulin gene and the calmodulin gene. Furthermore, the full coding sequence and promoter region of the *cyp51A*-gene was sequenced and microsatellite genotyping was performed [6]. Sequences were aligned with a reference cyp51A sequence (GenBank accession no. AF338659) to identify mutations. All isolates were stored in 10% glycerol at −80°C and subcultured on Sabauroud slants at 37°C.

Between 1970 and 2005 33 compounds were authorized by the Dutch Board for the Authorization of Plant Protection Products and Biocides for use as fungicides, herbicides, herbicide safeners and plant growth regulators, in The Netherlands. Of these 31 were available for testing including: amitrole, benomyl, biteranol, bromuconazole, carbendazim, cyazofamide, cyproconazole, difenoconazole, epoxiconazole, fenamidone, fenarimol, fenchlorazole-ethyl, fuberidazole, imazamethabenz-methyl, imazilil, metconazole, myclobutanil, nuarimol, paclobutrazole, penconazole, prochloraz, propiconazole, prothioconazole, pyrimethanil, tebuconazole, thiabendazole, thiophanate-methyl, triadimefon, triademinol I, triademinol II, triflumizole (Sigma Aldrich). The compounds were dissolved in DMSO and autosterilized for 30 minutes at room temperature. The minimal inhibiting concentration (MIC) was determined using a microbroth dilution format according to the CLSI M38-A2 reference method [17].

### Docking studies

The structure of wild type CYP51A protein *A. fumigatus* was derived from the crystal structure of human (PDB code: 3I3K) and *Mycobacterium tuberculosis* (Mt) (PDB code: 1EA1) lanosterol 14α-demethylase by homology modeling. Both proteins share 38% and 24% sequence identity with CYP51A of *A. fumigatus*, respectively and contain ligands in the active site bound to heme. The three-dimensional structures have been predicted by YASARA's homology modeling experiment (http://www.yasara.org). The experiment consists from building four models based on different alignment variants. The missing loops were modeled and optimizations of structures ware performed. The model with the best Z-score derived from the crystal structure of human lanosterol 14 α -demethylase was used for the presented studies.

In a recent publication by Fraczek et al. the *Mycobacterium* and human structures were also both compared and confirmed the choice for the human lanosterol 14 α -demethylase as the best template for the *A. fumigatus* model [18]. The structures of tested fungicides and medical triazoles (Table 1) were downloaded from PubChem (http://pubchem.ncbi.nlm.nih.gov/). We used FlexX for the docking experiment [19], [20]. The coordination of ligands to the iron atom of heme was treated as pharmacophore during the docking procedure. The water molecule present in the active site according to the crystal structure of 1EA1 was treated dynamically. The program checked automatically whether the presence of the water molecule had favorable contribution to the docking pose and only in such a case the water molecule was reported back, otherwise it was neglected. The flexibility of hydrogen atoms of Y107, Y121 and S297 was introduced to find an optimal docking pose for the ligand. Docking the respective compounds back into their crystal structure validated the docking procedure. The root mean square deviation (RMSD) of the positions for fluconazole (PDB code 1EA1) was 0.28 Å and for ketoconazole (PDB code 313K) 0.44 Å. All the binding modes present in the crystal structures were conserved [21], [22].

**Table 1:** Antifungal susceptibilities of medical triazoles and compounds used as fungicide, herbicide, herbicide safener and plant growth regulator.

Compound	Target site of action	Chemical group	Year	Median (Range) MIC50 (µg/ml)								Effect size r
				Clinical wild type		Environment wild type		Clinical TR/L98H		Environment TR/L98H		
Itraconazole	DeMethylation Inhibitors SBI: Class I	triazoles	1991	0.125	(0.063–0.5)	0.25	(0.125–1)	32	(4–32)	32	(16–32)	0.99
Voriconazole	DeMethylation Inhibitors SBI: Class I	triazoles	2001	0.5	(0.5–2)	0.5	(0.5–4)	4	(2–8)	4	(1–32)	0.82
Posaconazole	DeMethylation Inhibitors SBI: Class I	triazoles	2006	0.031	(0.016–1)	0.063	(0.031–0.25)	0.5	(0.25–1)	0.5	(0.25–0.5)	0.85
Carbendazim	Methyl Benzimidazole Carbamates	benzimidazoles	1973	2	(1–16)	8	(2–16)	4	(1–32)	4	(1–32)	0.17
Fuberidazole	Methyl Benzimidazole Carbamates	benzimidazoles	1973	32	(32)	32	(32)	32	(32)	32	(32)	0*
Thiabendazole	Methyl Benzimidazole Carbamates	benzimidazoles	1973	32	(32)	32	(16–32)	32	(16–32)	32	(32)	0.10
Benomyl	Methyl Benzimidazole Carbamates	benzimidazoles	1975	2	(2–8)	4	(2–16)	8	(2–32)	4	(2–32)	0.31
Thiophanate-methyl	Methyl Benzimidazole Carbamates	thiophanates	1975	32	(32)	32	(32)	32	(32)	32	(16–32)	0.01
Cyazofamid	Quinone inside Inhibitors	cyanoimidazoles	2002	32	(32)	32	(32)	32	(32)	32	(32)	0*
Imazalil	DeMethylation Inhibitors SBI: Class I	imidazoles	1978	0.125	(0.125–0.5)	0.25	(0.125–0.5)	2	(1–8)	2	(2–8)	0.94
Prochloraz	DeMethylation Inhibitors SBI: Class I	imidazoles	1987	0.5	(0.25–0.5)	0.5	(0.125–0.5)	1	(1–32)	1	(1–32)	0.51
Triflumizole	DeMethylation Inhibitors SBI: Class I	imidazoles	1992	8	(4–16)	8	(4–32)	32	(8–32)	32	(32)	0.87
Imazamethabenz-methyl	Acetohydroxyacid synthase inhibitors	imidazolinone	1993	32	(32)	32	(32)	32	(16–32)	32	(32)	0.00
Fenarimol	DeMethylation Inhibitors SBI: Class I	pyrimidines	1983	8	(8–32)	8	(8–32)	32	(16–32)	32	(32)	0.07
Nuarimol	DeMethylation Inhibitors SBI: Class I	pyrimidines	1993	16	(8–32)	16	(8–32)	32	(16–32)	32	(32)	0.84
Pyrimethanil	Methionine synthesis inhibitors	anilino- pyrimidines	1995	32	(32)	32	(32)	32	(32)	32	(32)	0*
Fenamidone	Quinone outside Inhibitors	imadazolinones	2005	32	(32)	32	(32)	32	(16–32)	32	(32)	0.00
Fenchlorazole	Acetyl CoA Carboxylase inhibitors	triazoles	1992	32	(32)	32	(32)	32	(32)	32	(32)	0*
Amitrole	DeMethylation Inhibitors SBI: Class I	triazoles	1970	32	(32)	32	(32)	32	(32)	32	(32)	0*
Triadimefon	DeMethylation Inhibitors SBI: Class I	triazoles	1980	32	(32)	32	(32)	32	(32)	32	(32)	0*
Bitertanol	DeMethylation Inhibitors SBI: Class I	triazoles	1983	4	(2–32)	16	(2–32)	32	(32)	32	(32)	0.71
Penconazole	DeMethylation Inhibitors SBI: Class I	triazoles	1986	32	(16–32)	32	(16–32)	32	(32)	32	(32)	0.36
Triadimenol I	DeMethylation Inhibitors SBI: Class I	triazoles	1988	32	(32)	32	(32)	32	(32)	32	(32)	0*
Triadimenol II	DeMethylation Inhibitors SBI: Class I	triazoles	1988	32	(32)	32	(32)	32	(32)	32	(32)	0*
Propiconazole	DeMethylation Inhibitors SBI: Class I	triazoles	1990	2	(2–4)	2	(2–8)	32	(16–32)	32	(16–32)	0.96
Cyproconazole	DeMethylation Inhibitors SBI: Class I	triazoles	1992	32	(8–32)	32	(2–32)	32	(16–32)	32	(16–32)	0.32
Tebuconazole	DeMethylation Inhibitors SBI: Class I	triazoles	1992	1	(1–4)	2	(1–8)	16	(8–16)	16	(8–16)	0.93
Myclobutanil	DeMethylation Inhibitors SBI: Class I	triazoles	1993	16	(8–32)	16	(4–32)	32	(32)	32	(32)	0.78
Difenoconazole	DeMethylation Inhibitors SBI: Class I	triazoles	1994	1	(1–2)	1	(1–4)	16	(8–32)	16	(8–16)	0.96
Epoxiconazole	DeMethylation Inhibitors SBI: Class I	triazoles	1994	2	(2–8)	2	(2–16)	32	(32)	32	(32)	0.96
Bromuconazole	DeMethylation Inhibitors SBI: Class I	triazoles	1996	1	(1–4)	1	(1–4)	16	(8–32)	16	(16–32)	0.95
Paclobutrazole	DeMethylation Inhibitors SBI: Class I	triazoles	1997	16	(8–32)	16	(8–32)	32	(16–32)	32	(32)	0.82
Metconazole	DeMethylation Inhibitors SBI: Class I	triazoles	2005	0.25	(0.125–0.5)	0.25	(0.125–0.5)	2	(1–4)	1	(1–2)	0.94
Prothioconazole	DeMethylation Inhibitors SBI: Class I	triazoles	2005	8	(2–16)	8	(2–16)	16	(8–32)	16	(16–32)	0.71

* Cannot be computed because at least one of the variables is constant.

### Microsatellite genotyping

Microsatellite genotyping was used to determine the genetic distances between TR_34_/L98H *A. fumigatus* isolates. A collection of 144 consecutive TR_34_/L98H isolates were used that originated from two prospective surveillance studies that were performed in the Netherlands. The first study included *A. fumigatus* isolates that were collected in Dutch hospitals between 1994 and 2007. A total of 1,912 *A. fumigatus* isolates were obtained from 1,219 patients from the Radboud University Nijmegen Medical Center [6]. In addition, 147 *A. fumigatus* isolates from 101 patients, from 28 other medical centers in the Netherlands were collected [4], [6]. The second culture collection included 1,792 *A. fumigatus* isolates that were collected from 1,192 patients in seven University Medical Centers in the Netherlands between 2007 and 2009 [8]. Both studies included an unselected collection of *A. fumigatus* isolates (clinically relevant as well as colonizing isolates) and used agar supplemented with itraconazole to detect for azole-resistance.

From six loci, consisting of three tri- and three tetranucleotide repeats, fragments were amplified by using fluorescently labeled primers. The sizes of the fragments were determined by addition of the GeneScan LIZ[500] marker and subsequent analysis of the fragments on the Applied Biosystems 3730 DNA analyzer. Assignment of repeat numbers in each marker was determined from the GeneScan data by using the Peak Scanner version 1.0 software (Applied Biosystems) [23]. By plotting the number of observed new genotypes versus the time on a semi-logarithmic scale, the year that the first new genotype emerged in The Netherlands was calculated with a 95% confidence interval by using the software package GraphPad Prism v5.00.

### Induction experiments

Induction experiments were performed with the medical triazole itraconazole (5 mg/l), the triazole DMIs bromuconazole (8 mg/l), difenoconazole (8 mg/l), epoxiconazole (16 and 32 mg/l), propiconazole (32 mg/l) and tebuconazole (8 mg/l) and all five DMIs combined together in concentrations ranging between 0.063–4 mg/l of each DMI. Wild type isolate CM237 and *akuB* ^KU80^ as well as recombinant *A. fumigatus* isolates *akuB* ^KU80^-TR3 containing the 34-bp tandem repeat and *akuB* ^KU80^-L98H2 containing the L98H substitution were used. A solution of 1×10^6^ of conidia was spread on a GYEP agar plate (glucose 2%, yeast extract 0,3%, peptone 1% and agar 2%) containing one or a combination of DMIs and subsequently passaged on GYEP agar slants with the same concentration of DMI(s). Agar plates and slants were incubated at 37°C, and isolate *akuB* ^KU80^-TR3 was also incubated at 25°C and 48°C. After 10 passages sequencing of the *cyp51A* promoter and full coding gene was performed to detect mutations.

### Statistical analysis

In order to express differences in MIC_50_ between wild type and TR_34_/L98H for the different compounds we first log transformed the MIC_50_ data and then computed point biserial correlations as correlation effect sizes (r) [24]. Values of r = 0 indicate similarity between MIC_50_'s and values of r = 1 indicate the largest relative dissimilarity. These correlation effect sizes cannot be computed in cases where all samples have identical MIC_50_ values, such as with compounds that show no *in vitro* activity against both wild type and TR_34_/L98H isolates. In those cases the correlation effect size was considered r = 0.

## Results

### Activity of fungicides against *A. fumigatus*

In the Netherlands 33 compounds have been authorized by the Dutch Board for the Authorization of Plant Protection Products and Biocides for use as fungicides, herbicides, herbicide safeners and plant growth regulators, between 1970 and 2005, of these 19 were DMIs (Table 1; Figure 1; Figure 2A). We were able to obtain 31 of these compounds as dry powder and investigated the *in vitro* activity against 38 TR_34_/L98H *A. fumigatus* isolates from clinical and environmental origin and 42 wild type controls. In addition, two azole-resistant isolates from environmental origin that harbor a transcriptional enhancer as a resistance mechanism and four isolates with point mutations in the *cyp*51A-gene that arose through patient therapy were also tested (Table 2). Differences in MIC_50_ between the wild type and TR_34_/L98H against all different compounds were computed as correlation effect sizes (r). The correlation coefficient is used as a measure of the size of an effect with a value of −1 indicating a negative correlation between the two variables, a value of 0 indicating no correlation and a value of 1 indicating a positive correlation. For the medical triazoles the effect sizes were 0.99 for itraconazole, 0.82 for voriconazole and 0.85 for posaconazole representing a positive correlation of dissimilarity between the MIC_50_'s of the wild type and TR_34_/L98H isolates. Dissimilarity between the MIC_50_'s was found for 20 compounds, with the greatest differences (r>0.90) found for propiconazole, difenoconazole, epoxiconazole (r = 0.96), bromuconazole (r = 0.95), metconazole (r = 0.94), imazalil (r = 0.94), and tebuconazole (r = 0.93) (Figure 2B). These compounds were DMIs from the triazole class, with the exception of imazalil. Isolates with a 46 bp or 53 bp tandem repeat insertion showed similar correlation effect sizes as TR_34_/L98H isolates (data not shown), while isolates that had become resistant through patient azole therapy generally showed lower r-values (Table 1) [25].

**Figure 1:** Chemical structures of antifungal compounds. Three medical antifungal compounds and 31 compounds that were authorized by the Dutch Board for the Authorization of Plant Protection Products and Biocides for use as fungicides, herbicides, herbicide safeners and plant growth regulators. The compounds are presented according to structural group.

**Figure 2:** Overview of introduction of the 31 compounds by year and correlation effect sizes. A) Overview of compounds by year of authorization by the Dutch Board for the Authorization of Plant Protection Products and Biocides (data from the Dutch Foundation for Phytofarmacy, Nefyto). The five triazole DMIs that exhibited the most identical docking by molecule alignment are underlined in blue. B) Correlation effect sizes (r) of compounds and medical triazoles comparing differences in the median MIC of wild type and TR_34_/L98H isolates. The fungicides are represented by grey dots and those belonging to the DMIs by black. The medical triazoles are indicated in red, and the five triazole DMIs that exhibited the most identical docking by molecule alignment are indicated in blue. *Correlation effect sizes could not be computed if in at least one of the two groups all variables were constant. This was the case with compounds that showed no *in vitro* activity against both wild type and TR_34_/L98H *A. fumigatus* isolates, and the correlation effect size was considered 0.

**Table 2:** Activity of medical triazoles and five DMIs against clinical and environmental *A. fumigatus* isolates with different *cyp*51A-mediated resistance mechanisms.

Resistance mechanism			Median MIC (mg/l)							
*cyp*51A gene*		# isolates	Medical triazoles&			DMIs				
Promoter region	Coding region		ITC	VCZ	POS	Bromuconazole	Difenoconazole	Epoxiconazole	Propiconazole	Tebuconazole
–	–	42	0.125	0.5	0.063	1	1	2	2	1
34 bp TR	L98H	38	>16	4	0.5	16	16	>16	>16	16
46 bp TR	Y121F, T289A	1	2	>16	0.5	>16	>16	>16	>16	16
53 bp TR	–	1	>16	16	0.25	16	>16	>16	>16	16
–	G54W	1	>16	0.25	>16	0.5	0.125	0.5	0.5	0.5
–	G54E	1	>16	0.25	1	0.25	0.25	0.5	0.5	0.5
–	M220I	1	>16	1	0.5	4	4	16	16	4
–	M220V	1	>16	2	1	4	2	8	4	4

* TR, tandem repeat.

& ITC, itraconazole; VCZ, voriconazole; POS, posaconazole.

### Molecule alignments and docking

We used a homology model of the *A. fumigatus* CYP-protein to predict the preferred orientation of DMI-compounds to form a stable complex with the 14α-lanosterol demethylase enzyme. A crystal structure of the *A. fumigatus* CYP51A protein is not available, therefore to see structural similarities in CYP51s for azole inhibition we superimposed the fluconazole-bound *Mycobacterium tuberculosis* (Mt) structure (PDB code 1EA1), the ketoconazole-bound human structure (PDB code 313K) and ketoconazole-bound *A. fumigatus* homology structure. Both fluconazole and ketoconazole bind to the heme iron via the nitrogen of an azole ring. The dihalogenated phenyl group, a common structural moiety of ketoconazole and fluconazole, occupied the same spaces at the active site of the heme molecule but interacts with the binding pockets lined by different residues when the human CYP51, the Mt CYP51 and the *A. fumigatus* CYP51 homology model are aligned. In human and *A. fumigatus* CYP51, residues Y145 and Y121, respectively formed van der Waals contacts with the dichlorophenyl group of ketoconazole, whereas their side-chain hydroxyl group made hydrogen bonds to the D-ring propionate (C_2_H_5_COO^−^) of the heme. Residue Y131 (PDB code 313K) that is located in the B′ helix of the homology structure (Y107) is invariant in the CYP51 family and involved in hydrogen-bond formation with heme A-ring propionate in all three structures. In the Mt structure, Y145-corresponding F89 is away from the active site due to the conformational flexibility of the B–C–helix region. Instead, R95 and R96 of Mt CYP51 are near the heme and fluconazole difluorophenyl group (Figure 3). Thus, ketoconazole could bind to Mt enzyme, utilizing the same space as fluconazole for the dihalogenated phenyl ring, while the remainder of ketoconazole would occupy the access channel observed in the human enzyme although the channel would have to be open by relocation of some of the side chains like F78 and M433 (grey structure Figure 3). In the Mt structure, the hydroxyl group of fluconazole made a water-mediated hydrogen bond to the heme A-ring propionate. This water molecule is not observed in the human structure because the cycle ether group of ketoconazole filled in the space of water. In addition, in Mt and *A. fumigatus* CYP51s an invariant H259/H296 residue from helix I is pointed into the active site, whereas the confirmation of the corresponding H314 in human CYP51 prevents its interaction with the inhibitors. The itraconazole, posaconazole and voriconazole molecules were docked into the *A. fumigatus* homology structure. They showed the same binding pattern as described for the crystal structures and were able to align to the presented poses of fluconazole (representative of voriconazole) and ketoconazole (representative of itraconazole and posaconazole). The compounds from the groups of imidazoles, pyrimidines and triazoles adopted similar poses upon docking in the active site of the *A. fumigatus* as those observed for the medical triazoles. The largest dissimilarities were in the cases of compounds that lack a phenyl group next to the 5- or 6-member aromatic ring that coordinates to the iron center. We performed a flexible alignment of the compounds on the structure of voriconazole in order to find the most similar compounds. The pharmacophores used as a filter for the alignment that consist of 5/6-member aromatic ring containing at least one nitrogen atom, a hydrogen-bond donor or acceptor and the aromatic functional group (Figure 4). The structures classified to groups of benzimidazoles, cyaninoimidazoles together with prochloraz, imazamethabenz from imidazolinone, and pyrimethanil from pyrimidines and fenamidone and amitrole from triazoles were filtered out from the set of the ligands as not similar to the voriconazole molecule. The remaining 20 of 31 structures were considered to be similar to the medical triazoles. We focused our analysis of the docking poses on the compounds that satisfied the given pharmacophores for alignment.

**Figure 3:** 3D representation of three aligned structures of CYP51 with the ligands in their active site, constructed by using the Yasara software. In green human CYP51 bound with ketoconazole from PDB: 3I3K; in gray Mt bound with fluconazole from PDB: 1EA1; in cyan *A. fumigatus* bound with ketoconazole from the homology model. The ligands are represented in balls and sticks, only the residues important for binding a particular ligand are depicted in the picture and represented in sticks. Numbering of the residues corresponds with their colors to the models.

**Figure 4:** Two-dimensional structure of voriconazole with indicated pharmacophores that were used to align and filter the 31 compounds (**Table 1**). The figure was constructed by using Marvin Sketcher form ChemAxon (www.chemaxon.com).

### Docking poses of fungicides similar to medical triazoles

The triazole DMIs that have three nitrogen atoms in the aromatic ring coordinated to the iron atom of heme made a hydrogen bond contact to residue S297, present in the active site of the *A. fumigatus* CYP51 homology model. Residue H296, also present in the active site, interacted with most of the fungicides with the exception of imazalil, triflumizole, fenarimol, nuarimol, penconazole, metconazole that instead interacted with a bridging water molecule. Propiconazole, myclobutanil, difenoconazole lack any interaction with residue H296 or a bridging water molecule. Most of the DMIs share the core structure with medical triazoles and due to this similarity they adopt much the same poses in the active site of *A. fumigatus* as the medical triazoles. Propiconazole and bromuconazole exhibit the most alike poses with the core structure being the most similar to itraconazole and posaconazole (Figure 5A). Tebuconazole and epoxiconazole also adopted the most alike poses being most similar to voriconazole, except they interacted with residue H296 in the active site (Figure 5B). The analysis of the top three poses proposed by the docking program showed that these compounds were able to adopt also poses where they interacted with a bridging water molecule instead of H296. This makes the binding modes of propiconazole, bromuconazole, tebuconazole and epoxiconazole most identical to those represented by the medical triazoles. Difenoconazole (Table 1) was different in structure from the rest of the cross-resistant DMIs. Instead of one aromatic ring (Figure 5A and 4B) it has a biphenyl moiety, upon docking this part was placed into the access channel where the long tail of medical azoles is normally located.

**Figure 5:** Analysis of most modes binding modes compared to the medical triazoles. A) Binding modes of propiconazole. This fungicide exhibits the most similar binding modes compared to the medical triazoles located in the active site of human and *A. fumigatus* CYP51. B) Binding modes of tebuconazole. This fungicide exhibits the most similar binding modes compared to the medical triazoles located in the active site of Mt CYP51. The main difference between A and B is the interactions with residue H296 in the active site, which is lacking in A.

The above mentioned five triazole DMIs were also among the compounds with the highest r-value and showed complete loss of *in vitro* activity against *A. fumigatus* isolates harboring TR_34_/L98H (Figure 2B, Table 1). Moreover, these five DMIs were authorized for use in the Netherlands between 1990 and 1996 (Figure 2A), which preceded the first known isolation of a clinical TR_34_/L98H isolate in 1998 [6]. Imazalil and metconazole also showed a high correlation effect size (Figure 2A), but, unlike the five abovementioned triazole DMIs, retained *in vitro* activity against TR_34_/L98H isolates (median MIC of 2 mg/l) (Table 1). Docking studies and molecule alignments showed that imazalil and metconazole were less similar to the medical triazoles and therefore less likely to have caused the emergence of TR_34_/L98H in *A. fumigatus*.

### Microsatellite genotyping

*A. fumigatus* isolates from two Dutch surveillance studies were used to investigate the evolution of TR_34_/L98H genotypes over time [6], [8]. The collections were obtained prospectively over a 16 year period and included 3,847 isolates from 2,512 patients. All isolates were screened for azole resistance by subculture on agar supplemented with itraconazole. The collections included 144 consecutive TR_34_/L98H isolates which were genetically characterized by short tandem repeat genotyping [23]. By plotting the number of observed new genotypes versus time on a semi-logarithmic scale, we calculated a rate of change of 1.37±0.05 genotype-1.year-1. Using the rate of change to calculate the year of first emergence of TR_34_/L98H, indicated that TR_34_/L98H had developed in the year 1997 (95% CI: 1993.7–1999.7) (Figure 6).

**Figure 6:** The evolution of new microsatellite genotypes over time based on short tandem repeat typing of 144 TR_34_/L98H *A. fumigatus* isolates, cultured between 1998 and 2009 in the Netherlands. By plotting the number of observed new genotypes versus time on a semi-logarithmic scale, a rate of change of 1.37±0.05 genotype-1.year-1 was calculated. As the first TR_34_/L98H isolate was cultured in 1998, the rate of change indicates that the first strain would have emerged around 1997 (95% CI: 1993.7–1999.7). This analysis also indicates that TR_34_/L98H had developed from a single ancestor.

### Induction of TR_34_/L98H

We investigated if the TR_34_/L98H substitutions could be induced during exposure to DMIs under laboratory conditions. A wild type *A. fumigatus* isolate and recombinants containing either the 34-bp insertion or the L98H substitution were exposed to itraconazole, bromuconazole, difenoconazole, epoxiconazole, propiconazole, tebuconazole or a mixture of these DMIs. The induction experiments generally resulted in a resistant phenotype within three passages. In three out of twelve clones of *A. fumigatus* cultured under itraconazole pressure, *cyp*51A-substitutions G138C or P216L were detected. These substitutions have been reported in patients who developed azole-resistant *Aspergillus* disease during itraconazole therapy [5]. TR_34_/L98H was not found in any of the clones that were exposed to itraconazole, single DMI compounds or to a mixture of DMIs. However, following exposure of the *A. fumigatus* conidia containing the 34-bp insertion in the *cyp51A*-gene promoter to 8 mg/l of tebuconazole resulted in one clone in which after three passages a triplicate of the 34 bp sequence was detected in the promoter region.

## Discussion

Although the hypothesis of a fungicide-driven route of azole resistance development in *A. fumigatus* is controversial [26], we provide evidence that such a route may exist. Five triazole DMIs were identified that exhibited very similar molecule characteristics to the medical triazoles, resulting in the most identical binding modes and the greatest level of cross-resistance. These five DMIs were authorized for use between 1990 and 1996, which was in keeping with our calculated date of origin of TR_34_/L98H based on microsatellite typing, and precedes the first clinical TR_34_/L98H isolate in 1998. Continued triazole DMI pressure and lack of an apparent fitness cost in TR_34_/L98H isolates are probably important factors that have facilitated the ability of TR_34_/L98H to sustain in the field in competition with wild type isolates.

Although the relation between the use of antimicrobial agents outside human medicine and the development of resistance to clinically used compounds has been shown for bacteria, we show for the first time evidence that the same principle may occur in molds. Culture-based surveillance studies increasingly report TR_34_/L98H in clinical and environmental isolates in Europe and, most recently, in China [14]. Moreover, there is very recent evidence that two new ‘environmental’ azole resistance mechanisms have emerged in *A. fumigatus* in the Netherlands, of which one has rapidly migrated across the country similar to TR_34_/L98H [27]. However, surveillance studies based on positive cultures may underestimate the prevalence of resistance. Detection of azole resistance mechanisms directly in clinical specimens from patients with chronic lung diseases showed that in culture-negative, PCR-positive samples *cyp51A*-mutations were detectable in as many as 55.1% of respiratory samples [28]. These observations indicate that we are just beginning to understand the scale of the problem, but it suggests that azole resistance in *A. fumigatus* has become a public health problem and threatens an increasing population of (immunocompromised) patients.

Our study was limited by the fact that we were unable to induce the full TR_34_/L98H resistance mechanism during DMI-pressure under laboratory conditions, using an isolate that is deficient in DNA break repair. Previously, microsatellite genotyping showed shorter genetic distances for TR_34_/L98H isolates compared with wild type isolates [10], which suggests that TR_34_/L98H isolates may have originated from a common ancestor. If this would be the case, the development of TR_34_/L98H would be extremely infrequent in the environment and would explain why we were unable to induce TR_34_/L98H under laboratory conditions. However, this may point to other reasons for the emergence of TR_34_/L98H. TR_34_/L98H isolates may have other properties, such as increased fitness or virulence, or high sporulation efficacy, that have made isolates harboring TR_34_/L98H more successful in the field than wild type *A. fumigatus*. However, at present there is no evidence that supports increased virulence in TR_34_/L98H isolates. Animal studies indicate that the virulence of TR_34_/L98H is similar to that of wild type isolates, although only one TR_34_/L98H isolate was used [3]. An alternative explanation for our inability to induce TR_34_/L98H could be that this resistance mechanism developed through sexual or parasexual reproduction rather than asexual reproduction, which was not tested in the laboratory. However, we did observe one isolate in which two copies of the tandem repeat evolved into three, supporting the role of DMIs in inducing genomic changes in cyp51A of *A. fumigatus*. Another limiting factor of our studies was the lack of sequence-based evolutionary analysis. In *A. fumigatus* no genes have been described that are suitable for this type of analysis and therefore we used microsatellite data.

The relation between the use of the triazole DMIs and cross-resistance to medical triazoles in *A. fumigatus* has major implications for the assessment of health risks associated with the use of DMIs. Molecule structure similarity and activity of triazole DMIs against *A. fumigatus* appear to be the key features that cause cross-resistance to medical triazoles. Further research should be aimed at understanding the conditions under which resistance mechanisms develop in the environment and which *Aspergillus* morphotype is most prone to develop resistance mechanisms. Reversal of resistance development may be achievable by restriction of certain triazole DMIs, but laboratory population studies and genetic mapping would be required to predict the impact of changes in DMI-pressure. In addition, there is limited insight in the use of fungicides for agricultural and non-agricultural applications.

The continued use of DMIs with activity against opportunistic human fungal pathogens is a risk for the management of fungal diseases caused by these pathogens. The number of classes of drugs available for treating non-invasive and invasive fungal diseases is limited and the triazoles are the only class of antifungal agents that can be administered orally. A fungicide-driven route of resistance development in TR_34_/L98H could indicate that such mechanisms may also occur in other *Aspergillus* species or other opportunistic fungi. It is therefore of great importance to perform abovementioned research as it may allow the implementation of evidence-based strategies aimed at elimination of the fungicide-driven route of azole resistance development in opportunistic fungi.
